The article "Knowledge-Based Discovery of the Role and Mechanism of Resveratrol in Improving Glomerular Tether Cell Proliferation and Apoptosis in Diabetic Nephropathy" was retracted in 2023. Reasons: signs of a paper mill; suspected computer-generated content; unreliable results or conclusions; lack of ethics approval or compliance.

# Knowledge-Based Discovery of the Role and Mechanism of Resveratrol in Improving Glomerular Tether Cell Proliferation and Apoptosis in Diabetic Nephropathy

**DOI:** 10.1155/2022/9705144

**Published:** 2022-03-31

**Authors:** Yangfeng Chi, Shuang Liu, Xinye Wu, Bingbing Zhu, Hao Wang, Yongping Liang, Yunman Wang

**Affiliations:** Department of Nephrology, Putuo Hospital, Shanghai University of Traditional Chinese Medicine, ShangHai 200062, China

## Abstract

To investigate the effects and mechanisms of resveratrol on glucolipid metabolism in diabetic humans. In this paper, we introduced the knowledge discovery theory into the data processing of the factors related to the pathogenesis of type 2 diabetes for the first time, and identified valid, potentially useful, and understandable pathogenesis patterns from a large amount of measured data. A data mining C4.5 algorithm was used to classify 17072 validated cross-sectional health survey data from the whole population according to the characteristics of type *ρ* diabetes data. A human model of diabetes mellitus was prepared by high sugar and high fat diet plus low dose streptozotocin (STZ, 35 mg/kg) and randomly grouped into four groups: the normal control group, the model group, the resveratrol group, and the pioglitazone group. 8 animals in each group were treated with the corresponding drugs for 8 weeks. Hepatic steatosis and damage were significantly reduced compared with the model group as observed by HE staining. Resveratrol has obvious effects on regulating glucolipid metabolism, and its mechanism of action is associated with its ability to increase the antioxidant activity of the body, activate the Akt signaling pathway, and improve liver pathological damage.

## 1. Introduction

With socioeconomic progress and development, the spectrum of diseases that threaten human health is changing. Chronic noncommunicable diseases are a growing threat to the health of the population, especially the elderly, and most notably, the prevalence of type 2 diabetes mellitus is on the rise in a near epidemic worldwide. Type 2 diabetes mellitus occurs due to a combination of genetic and environmental factors, and the interplay of these factors is complex [1]. Many factors associated with the onset of diabetes have been proposed by applying current research tools, but it is difficult to establish further linkages and identify patterns among these factors. In the face of the limitations of traditional statistical studies with huge and complex data, this paper attempts to investigate this problem through bioinformatics. Knowledge discovery is one of the main techniques in bioinformatics. It is an advanced process of identifying valid, potential, and understandable patterns from large amount of data and is a class of deep data analysis methods [2, 3]. It can extract the regular content hidden behind the data from large-scale data and is widely used in decision support and scientific research. Based on the database and data preparation, we introduced the knowledge discovery theory into the data processing of type 2 diabetes, and used the data mining C4.5 algorithm to automatically build a decision classification tree according to the characteristics of the data. The system was trained to identify the relationship between the prevalence factors of type 2 diabetes and determine whether the disease was present [4, 5]. The application of this algorithm laid the foundation for further exploration of the pathogenesis of type 2 diabetes and the development of disease prediction models.

GSK-3*β* is a key enzyme involved in hepatic glucose metabolism, inhibiting its activity by phosphorylating glycogen synthase, decreasing hepatic glycogen synthesis and increasing blood glucose concentration in the body, with abnormally high expression in diabetic and obese humans [6]. -3*β* is a downstream signaling molecule directly regulated by Akt, and when the upstream Akt signaling molecule is activated, GSK-3*β* is inhibited, preventing its inhibition of hepatic glycogen synthesis and thus facilitating the conversion of glucose uptake by the body after meals. Inhibition of GSK-3*β* activity plays a crucial role in glycogen synthesis [7, 8].

Hepatic glycogen is the main form of glucose storage in the body, and the body converts excess glucose in the blood into glycogen stored in the body through a series of enzymatic reactions mediated by signaling pathways, thus reducing blood glucose concentration. Therefore, increased hepatic glycogen synthesis facilitates the reduction of hepatic glycogen output for the purpose of lowering blood glucose. The experimental results showed that resveratrol could promote hepatic glycogen synthesis and lower blood glucose levels by increasing Akt phosphorylation activity, inhibiting downstream GSK-3*β* phosphorylation activity, and promoting downstream GCK protein levels in diabetic model animals [9, 10]. It is suggested that resveratrol may achieve the effect of lowering blood glucose by upregulating Akt activity.

Diabetic fatty liver is a common and frequent chronic complication that seriously endangers the health of diabetic patients during the onset, development, and treatment of diabetes. Some clinical studies have confirmed that liver lesions can be as high as 46% in diabetic patients. Patients who develop fatty liver can further aggravate the pathological conditions such as insulin resistance and glucose metabolism disorders, which in turn promote the deterioration of diabetes. Abnormal liver function, which affects the normal glucose metabolism function and the inability to convert excess blood glucose into hepatic glycogen for storage, can result in persistently high blood glucose levels and aggravate diabetes [11, 12]. Resveratrol can significantly regulate the body's disorders of glucose and lipid metabolism, improve the body's antioxidant activity, delay liver damage, and improve the formation and development of diabetic complications. Resveratrol has obvious antioxidative stress effects and can avoid oxidative stress damage induced by high sugar and high fat, thus playing an important role in the prevention and treatment of diabetes and its chronic complications, especially in the early stages of diabetes to delay the development of diabetic complications and protect other organ tissues. It can play an important role in the prevention and treatment of diabetes and its chronic complications, especially in the early stages of diabetes to delay the development of diabetic complications and protect other organ tissues [13–15]. Resveratrol is a natural drug with great potential, and the prospect of clinical application needs further study.

## 2. Data Sources, Scale, and Preprocessing Methods

The measured data were obtained from a cross-sectional survey of a whole cohort sample of 17,946 people in our hospital, from which 17,072 valid data were selected. Each data record was divided into five sections: general personal data, living and working habits, past and family medical history, physical examination data, and laboratory test data. The investigators who participated in the data collection were trained in a standardized way and used a standardized questionnaire to collect personal data; life and work habits; and medical history to determine height, weight, abdominal circumference, and blood pressure by a standardized method. Blood glucose and lipids (cholesterol, triglycerides, LDL, and HDL) were measured in a strictly quality-controlled laboratory. The diagnostic criterion for diabetes mellitus was fasting blood glucose >7.0 mmol/l [16].

The abovementioned raw data were entered into the computer and a database was established. Raw data preprocessing was used to improve the quality of the data for incomplete, noisy, and inconsistent raw data, and thus improve the quality of the excavation results. The data preprocessing process used in this paper mainly includes data cleaning, data transformation, and data statute (the specific method is published in a separate paper). The data (11,400 items) were randomly extracted from the preprocessed data by the C4.5 algorithm as the training data of the C4.5 algorithm, and the rest of the data were used as the test data. The operating system is Solaris8, and the C++ compiler is c.

In order to make the program run on the laris platform, a Makefile file for the Solaris platform was written in addition to the ANSI C implementation. After compiling and linking with cc, the executable version for the Solaris platform is generated.

## 3. Choice of Algorithm

The data in this paper are characterized by the predictive and continuous nature of the classifications, and it is known whether each set of data corresponds to a classification of diseased or undiseased data. The main task of this paper is to learn the classification patterns in the data. Based on the categorical nature of the mining task, the decision tree algorithm, which is least affected by the record fields, easy to understand the model, easy to train the model, easy to implement the model, has the most generality, and highest usefulness, was selected for mining. The C4.5 algorithm is a very effective decision tree algorithm, which can handle continuous data items. Therefore, the C4.5 algorithm is the preferred algorithm for data mining in this work [17].

## 4. C4.5 Principle of the Decision Tree Classification Algorithm

C4.5 is an algorithm for constructing decision tree classifiers, which is an extension of the ID3 algorithm. While the I3 algorithm can only handle discrete descriptive attributes, the C4.5 algorithm can also handle cases where the descriptive attributes are continuous. This algorithm uses a comparison of the magnitude of the information gain value of each descriptive attribute to select the attribute with the largest gain value for classification. If there are continuous descriptive attributes, then the values of these continuous attributes are first divided into different zones, i.e., “discretized”. The method of “discretizing” continuous attributes is as follows:

(1) $$\begin{array}{c} A_{i}=\text{MIN}+\frac{\text{MAX}-\text{MIN}}{N}\times i,\;i=1,2,\ldots ,N. \end{array}$$

AK, the largest F57C value, is selected as the breakpoint for this continuous attribute, and the attribute value to [MIN,AK] and (AK, MAN) interval values is set[18].

(2) $$\begin{array}{c} S=-\sum_{I}\left(p_{i}^{*}\log\left(p_{i}\right)\right). \end{array}$$

The information gain described in the paper is the effective reduction of information entropy, according to which it is possible to determine what variables at what level to classify the algorithm in the application by two processes a training process to derive the classification algorithm, and a testing process, i.e., to derive the correct recognition rate. The experiment is to select about two-thirds of the 17072 valid data, i.e., 11400 as training data and the remaining 5672 as test data.

## 5. Case Study

### 5.1. General Materials

Healthy Wistar male rats, SPF class, 50 rats, body weight (120 ± 15) g, were purchased from the Guangdong Experimental Animal Center, and the experiments were performed in an SPF class laboratory at 20–25°C, 40%–70% relative humidity, and 10–15 air changes/h. Resveratrol (purity = 95.1%, HPLC) was provided by Shaanxi Saide Hi-Tech Biological Co. Ltd. High-fat and high-sugar feed formula: 0.5% bile salt, 1% cholesterol, 1% egg yolk powder, 10% lard, 20% sucrose, 67.5% common feed.

### 5.2. Main Reagents

Trace malondialdehyde (MDA), liver glycogen, and other measurement kits were purchased from Nanjing Jiancheng Institute of Biological Engineering; concentrated sulfuric acid (AR) was purchased from Guangzhou Chemical Reagent Factory; p-Akt, p-GSK-3*β*, GSK-3*β*, and GAPDH antibodies were purchased from Cell Signaling, USA; Akt and GCK antibodies were purchased from Santa Cruz, USA; and streptozotocin (STZ) was purchased from Sigma, USA.

### 5.3. Results

Compared with the normal group, the diabetic humans showed the typical symptoms of diabetes, such as fasting blood glucose, serum TC, TG, and LDL-C levels, and the difference was statistically significant (P＜0.05). After 8 weeks of treatment, the symptoms of “three more and one less” in all diabetic groups were improved, and the levels of fasting blood glucose, TC, TG, and LDL-C were significantly reduced, and the levels of HDL-C were increased in each group, and the difference was statistically significant (P＜0.05) [19]. It is suggested that resveratrol has the effect of lowering blood glucose and also has a certain effect on lipid regulation (Table 1).

The liver of the model group showed a significant decrease in liver glycogen content compared with the normal group, and the difference was statistically significant (*P* < 0.05). In the resveratrol and pioglitazone groups, the liver glycogen content increased significantly compared with the model group, and the difference was statistically significant (*P* < 0.05) [20]. This suggests that resveratrol has the effect of significantly increasing the liver glycogen content and promoting the storage of glycogen in the body, which not only promotes the utilization of blood sugar but also plays an important role in preventing the occurrence of multiorgan complications in the body (Figure 1).

The level of SOD activity reflects the ability of the body to scavenge oxygen free radicals, while the level of MDA content reflects the severity of free radical attack on the body cells. The results of SOD activity and MDA content were used to analyze the ability of the organism to resist oxygen stress. In the model group, SOD activity decreased and MDA content increased compared with the normal group, and the difference was statistically significant (*P* < 0.05); in the drug administration group, SOD activity increased and MDA content decreased compared with the model group, and the difference was statistically significant (*P* < 0.05) [21]. The effect of the resveratrol group has significantly improved the level of oxidative stress in the body, thus controlling the occurrence of diabetic complications (Figure 2).

The protein expression of phosphorylated Akt was significantly reduced in the model group rats relative to total Akt, and the phosphorylated expression of Akt protein was inhibited, while resveratrol and pioglitazone could effectively increase the phosphorylated expression level of Akt protein in the livers of model animals (Figure 3).

The active form of GSK-3*β* in the model group, phosphorylated-GSK-3*β* relative to total-GSK-3*β* protein expression level, was significantly higher than that in the normal group, and the difference was statistically significant (*P* < 0.05). The resveratrol group could significantly reduce the protein expression of p-GSK-3*β* compared with the model group, and the difference was statistically significant (*P* < 0.05), suggesting that resveratrol could effectively inhibit the phosphorylated expression level of GSK-3*β* protein in the liver (Figure 4).

The protein expression level of glucokinase in the model group was significantly decreased compared with the normal group, and the difference was statistically significant (*P* < 0.05). The resveratrol group could significantly increase the protein expression of GCK in the diabetic human liver, and the difference was statistically significant (*P* < 0.05). The difference was statistically significant (*P* < 0.05) [22], suggesting that resveratrol could effectively increase the protein expression level of GCK in the diabetic human liver based on the activation of liver Akt protein phosphorylation expression (Figure 5).

In the resveratrol group, the morphology of hepatocytes was normal, the nuclei were clear, small lipid droplets were still visible in the plasma of some hepatocytes, and the boundaries of local cells were unclear. The hepatocyte cords were arranged neatly and radially, the hepatic sinusoids were normal, and some of the hepatic cords were disordered. The degree of hepatic steatosis and damage was significantly reduced compared with that of the hyperlipidemic diabetic human model group. In the pioglitazone group, the degree of hepatic steatosis and damage was reduced compared with that in the hyperlipidemic diabetic human model group, but a large number of fat vacuoles of different sizes and uneven cytoplasmic staining were still visible in the hepatocytes (Figure 6).

## 6. Experimental Results

By using the C4.5 algorithm, the following decision classification tree was derived, where N indicates no disease and Y indicates disease (the main reason for giving this type of classification decision tree is that the values in the classification can be directly observed, such as the blood glucose value (GLU) of 5.85, as the threshold value of the main classification is very important, the value tends to be consistent with the medical understanding), as shown in Figure 7.

As shown in Figure 7, a total of 31 nodal parameters entered into the decision tree accounted for 66% of all investigated parameters, classified according to the larger information gain value (information gain value) determined by this algorithm. Among them, there were 10 node parameters in the first 5 levels, including age, family history of diabetes, dietary habits, hyperlipidemia, etc. The nodal parameters in the first 10 levels were 30, including abdominal circumference, body weight, blood pressure, and lipids. The composition of these parameters tended to be consistent with the known risk factors in medicine, especially the threshold value of 5.85 for the classification of blood glucose, which is of great importance for the classification of risk factors of diabetes in medicine. Finally, the classification accuracy was tested by randomly dividing the given data into two independent sets, i.e., the training set and the test set, and specifically, 5672 test samples were used in the experiment, including 340 diseased samples.

As shown in Figure 8, this is consistent with the domestic report of Geng [4], and also with the foreign study of Young et al. [3] in diabetic rats in vivo. And they found that the cause of the proliferation of diabetic glomerular tract cells was related to the paracrine secretion of PDGF and bFGF. In contrast, studies in the commonly used high glucose model (normal glomerular thylakoid cells in culture stimulated by high glucose) showed that high glucose promoted ECM secretion but inhibited MC proliferation. This suggests that a brief high glucose stimulation (a few days) cannot mimic the glomerular thylakoid cells in vivo (there are other pathogenic factors besides high glucose, and it is a chronic pathological process), which also suggests that a diabetic model followed by MC culture is a good way to study glomerular thylakoid cells in DM.

## 7. Conclusions

The common approaches to knowledge discovery mainly include techniques such as artificial neural networks, decision trees, genetic algorithms, nearest neighbor algorithms, rule derivation, fuzzy theory methods, and visualization. Although almost all data mining techniques can be described as data-driven rather than user-driven, i.e., the user only needs to give the data when using these algorithms and does not have to tell the algorithm what to do and what results to expect; everything is found by the algorithm itself from the given servant data. Based on the ID3 algorithm, a variety of decision tree algorithms have been developed, and the C4.5 algorithm is one of them. It is an extension of the I3 algorithm.

## Figures and Tables

**Figure 1:** Effect of liver glycogen content in liver tissue.

**Figure 2:** Effect of resveratrol on SOD activity and MDA content in diabetic human serum.

**Figure 3:** Effect of resveratrol on the phosphorylation level of Akt in diabetic human liver.

**Figure 4:** Effect of resveratrol on GSK-3*β* activity in diabetic humans.

**Figure 5:** Effect of resveratrol on diabetic human glucose kinase (GCK) protein expression.

**Figure 6:** HE staining of human liver tissue in each group.

**Figure 7:** Clustering subcases of different methods.

**Figure 8:** Recognition efficiency.

**Table 1:** Comparison of glycolipid metabolic indexes in each group after drug administration and treatment ($\bar{x}\pm s$, *n* = 8).

Group	FBG	TC	TG	LDL-C	HDL-C
Normal group	4.52 ± 0.44	1.32 ± 0.19	0.73 ± 0.25	0.27 ± 0.13	0.59 ± 0.04
Model group	24.6 ± 2.31	12.1 ± 0.68	3.48 ± 0.43	7.13 ± 3.65	0.54 ± 0.2
Resveratrol group	14.3 ± 3.4	2.71 ± 0.41	1.08 ± 0.31	0.75 ±.33	0.81 ± 0.12
Pioglitazone group	13.6 ± 3.01	2.42 ± 0.52	0.92 ± 0.49	0.69 ± 0.15	0.91 ±.13

## Data Availability

The data underlying the results presented in the study are available within the manuscript.
